# Cancer Stem Cells: Emerging Key Players in Immune Evasion of Cancers

**DOI:** 10.3389/fcell.2021.692940

**Published:** 2021-06-21

**Authors:** Martina Mang Leng Lei, Terence Kin Wah Lee

**Affiliations:** ^1^Department of Applied Biology and Chemical Technology, The Hong Kong Polytechnic University, Kowloon, Hong Kong; ^2^State Key Laboratory of Chemical Biology and Drug Discovery, The Hong Kong Polytechnic University, Kowloon, Hong Kong

**Keywords:** cancer, cancer stem cells, immune cells, tumor microenvironment, immune evasion

## Abstract

Cancer stem cells (CSCs) are subpopulations of undifferentiated cancer cells within the tumor bulk that are responsible for tumor initiation, recurrence and therapeutic resistance. The enhanced ability of CSCs to give rise to new tumors suggests potential roles of these cells in the evasion of immune surveillance. A growing body of evidence has described the interplay between CSCs and immune cells within the tumor microenvironment (TME). Recent data have shown the pivotal role of some major immune cells in driving the expansion of CSCs, which concurrently elicit evasion of the detection and destruction of various immune cells through a number of distinct mechanisms. Here, we will discuss the role of immune cells in driving the stemness of cancer cells and provide evidence of how CSCs evade immune surveillance by exerting their effects on tumor-associated macrophages (TAMs), dendritic cells (DCs), myeloid-derived suppressor cells (MDSCs), T-regulatory (Treg) cells, natural killer (NK) cells, and tumor-infiltrating lymphocytes (TILs). The knowledge gained from the interaction between CSCs and various immune cells will provide insight into the mechanisms by which tumors evade immune surveillance. In conclusion, CSC-targeted immunotherapy emerges as a novel immunotherapy strategy against cancer by disrupting the interaction between immune cells and CSCs in the TME.

## Introduction

Cancer stem cells (CSCs) are subsets of cancer cells enriched with stem cell-like characteristics, including self-renewal ability and multilineage differentiation (Bhatia and Kumar, 2016). The CSC theory of tumor progression presents the tumor microenvironment (TME) as a hierarchically organized tissue with a CSC subpopulation ranked at the top level, which generates more differentiated cancer cells with lower or limited proliferative potential. CSCs are often defined by the expression of surface stem cell markers such as CD24, CD34, CD44, CD47, CD133, and CD90, along with side populations that can be isolated and enriched *in vitro* and *in vivo* without stem cell surface markers (Taniguchi et al., 2019). Epithelial-to-mesenchymal transition (EMT) is well known to be an inducer of CSC phenotypes via epigenetic regulation (Bocci et al., 2019). Its activation allows CSCs to drive resistance to conventional therapy and thus leads to treatment relapse and tumor reoccurrence (Shibue and Weinberg, 2017).

A substantial body of literature has extensively described the interactions of tumor bulks with the immune system; however, investigations have only begun to elucidate the relationship of CSCs and immune cells within the TME, paving the way for the development of rational therapeutic strategies to explore CSC-immune dynamics. The capability of CSCs in tumor initiation in partly immunocompromised mice e.g., SCID or NOD/SCID mice (T, B cells defect but NK cells present) suggests that these cells are empowered with the definitive ability to evade immune detection and surveillance, whereas non-CSCs require a higher extent of deficiency in immune system for generating tumors in NSG mice (lack of T, B, and NK cells) (Tsuchiya and Shiota, 2021). Increasing evidence has demonstrated that there is a reciprocal interaction between CSCs and various immune cells. Major immune cells within the TME drive CSC expansion and concurrently elicit protumorigenic immune cell activities, promoting CSC-specific avoidance of immune detection and destruction. In this section, we will discuss the emerging knowledge of the role of tumor-associated macrophages (TAMs), dendritic cells (DCs), myeloid-derived suppressor cells (MDSCs), T regulatory (Treg) cells, natural killer (NK) cells, and tumor-infiltrating lymphocytes (TILs) in driving cancer stemness and how CSCs evade the immune surveillance of these cells. Finally, we will discuss the potential of CSC-targeted immunotherapy to eradicate cancer.

## Tumor-Associated Macrophages

Macrophages can be classified into two subtypes: pro-inflammatory M1 and anti-inflammatory M2 macrophages (Chen et al., 2019). TAMs usually express an M2 phenotype, which executes immunosuppressive and pro-tumor functions and is thus closely related to cancer progression and recurrence (Lewis and Pollard, 2006; Malfitano et al., 2020).

Developing findings support the hypothesis that CSCs influence the immune TME via the recruitment of macrophages and the promotion of their pro-tumor properties, while TAMs, in turn, are crucial for the self-renewal ability and maintenance of CSCs in primary tumors through the coupling between STAT3 and NF-κB signaling cascades (Sainz et al., 2016). It has been proposed that CSCs have an intrinsic immunosuppressive program involving recruiting macrophages and driving them toward M2 polarization at the tumor site (Brissette et al., 2012). This ability of CSCs is commonly found in ovarian, glioblastoma, liver, breast and lung cancers through activating the signal transducer and activator of transcription 3 (STAT3) and nuclear factor-κB (NF-κB) pathways and cytokines such as interleukin (IL)-8 and IL-10 (Iliopoulos et al., 2009; Ginestier et al., 2010; Mitchem et al., 2013; Fang et al., 2014). For example, in hepatocellular carcinoma (HCC), CD133^+^ cells induce M2 polarization of TAMs through secretion of IL-8 (Xiao et al., 2018). In glioblastoma, CSCs generate higher levels of the chemoattractants C-C motif chemokine ligand 2 (CCL2), CCL5, vascular endothelial growth factor-A (VEGF-A), and neurotensin than the bulk of the glioma (Yi et al., 2011). The extracellular matrix protein periostin is preferentially expressed on CD133^+^CD15^+^ glioma CSCs and recruits macrophages through integrin αvβ3 from the peripheral blood to the brain (Zhou et al., 2015). Depletion of periostin in glioma CSCs leads to a reduction in the M2 population and alleviates tumor growth in glioblastoma xenografts. In breast cancer, Sox2^+^ cancer cells, via activation of nuclear factor of activated T-cells (NFAT), STAT3 and NF-*κ*B, express chemokines CCL3 and ICAM-1 and thus recruit TAMs into the TME (Yang et al., 2013; Mou et al., 2015). These findings suggest that CSCs play an important role in TAM recruitment and M2 polarization by secreting macrophage chemoattractants.

Subsequent to TAM recruitment to the TME, TAMs are deployed as a “niche” to support CSC growth. Infiltrating TAMs, by activating the NF-κB signaling pathway, secrete the inflammatory cytokines IL-1β, IL-6, IL-10, transforming growth factor beta (TGF-β), and MFG-E8 (Jinushi et al., 2011; Li et al., 2012; Fang et al., 2014; Wan et al., 2014; Yang et al., 2019). These tumor-promoting cytokines bind to their receptors, further stimulating STAT3 activation in adjacent CSCs. This results in a vicious cycle of NF-κB activation as well as stemness maintenance of cancer cells. For example, treatment of breast cancer cells with conditioned medium of TAMs leads to increments in the stem cell markers Sox-2, Oct3/4 and Nanog with enhanced ALDH1 activity in a mouse model (Nnv and Kundu, 2018). The abrogation of STAT3 confirmed the role of JAK/STAT pathway in mediating TAM regulation on CSC enrichment. In coculture systems, recruited TAMs promote liver CSC expansion through IL-6/STAT3, Wnt/β-catenin and TGF-β signaling pathways (Fang et al., 2014; Wan et al., 2014; Chen et al., 2019). TAMs preferentially secrete TGF-β to stimulate CSC-like properties by inducing EMT, while TAM-derived IL-6 induces CD44^+^ HCC stem cell expansion by activating STAT3, thus promoting tumor development through CSC growth. Blockade of IL-6 with tocilizumab and STAT3 knockdown attenuated CD44^+^ sphere formation and tumor growth of patient-derived HCC as well as breast xenografts (Wan et al., 2014; Wang et al., 2018a).

To facilitate communication, TAMs establish direct adhesion with CD90^+^ CSCs through EphA/ephrin A signaling and promote tumor initiation in breast cancer tissue (Lu et al., 2014). The EMT program first induces the expression of the surface ligands Thy1 and EphA4, which enable more frequent cell-cell interactions between TAMs and CSCs. Upregulated TAM-CSC contact thus activates the EphA4 receptor on CSCs and its downstream Src and NF-κB pathways (Iliopoulos et al., 2009; Lu et al., 2014). NF-κB activation positively reinforces the secretion of cytokines, including IL-6, IL-8, and GM-CSF, which are crucial for CSC self-renewal and stemness state maintenance (Rinkenbaugh and Baldwin, 2016; Choi et al., 2019). Interestingly, proinflammatory M1 macrophages were also found to play a role in breast CSC formation due to their activation of the STAT3 and NF-κB pathways by CD44^*high*^/CD24^–/low^ or ALDH1^+^ CSCs, while M2 macrophages maintained a higher population of ALDH^+^ cells (Guo et al., 2019). There is a possibility that M1 macrophages, through M2-mediated signaling, modulate CSC formation and regulate tumor initiation. Other signaling pathways, such as PTN/β-catenin, Notch1 and p38-MAPK, are also involved in stimulating CSC self-renewal in lymphoma, lung and ovarian cancers via the preferential secretion of IL-10 and IL-17 by TAMs (Xiang et al., 2015; Wei X. et al., 2019; Yang et al., 2019). Taken together, TAMs, through activating STAT3 and NF-κB signaling cascades and cytokines IL-1β, IL-6, IL-8, IL-10, and IL-17 and growth factor TGF-β, play an important role in the self-renewal and chemoresistance of CSCs.

Numerous studies have demonstrated the direct regulation of CSC self-renewal and proliferation by TAMs. CSCs also take advantage of TAM immunosuppressive functions to escape immune surveillance. In HCC, TAMs provide a “safe” environment for CSCs by overexpressing SIPRα, which interacts with CD47 that in turn acts as a “Don’t eat me” signal and protects CSCs from being phagocytosed. Recently, CD24, one of the liver CSC markers, was identified to be another “Don’t eat me” signal to macrophages by binding to inhibitory receptor sialic-acid-binding Ig-like lectin 10 (Siglec-10) (Lee et al., 2014; Barkal et al., 2019). Liver CSCs may also escape the clearance of macrophages by interacting with their surface Siglec-10 receptor. TAMs also influence T-cell cytotoxic activity by stimulating immune checkpoint molecules such as programmed death-ligand 1 (PD-L1) in cancer cells and T cell immunoglobulin and mucin domain-containing protein 3 (TIM-3), programmed cell death protein-1 (PD-1) and cytotoxic T-lymphocyte-associated protein-4 (CTLA-4) on the T cell surface, leading to an impaired immune response (Cassetta and Kitamura, 2018; Liu et al., 2018; Xiao et al., 2018). Interestingly, it has been proposed that leukemic CSCs secure their survival by overexpressing TIM-3, which promotes MDSCs and subsequent differentiation into TAMs in the leukemic stem cancer niche (Kikushige et al., 2010; Gao et al., 2014; Raggi et al., 2016). The relationship between TIM-3 expression and CSCs has also been shown in melanoma, osteosarcoma, as well as liver, lung, and ovarian cancers (Fourcade et al., 2010; Gao et al., 2012). To protect themselves from being targeted, deterioration in the antigen-presenting ability of TAMs also minimizes macrophage stimulation of T-cell and NK cell cytotoxicity activity (Lewis and Pollard, 2006).

In summary, complicated STAT3/NF-*κ*B crosstalk is established between CSCs and TAMs in the TME, in which CSCs attract, re-educate, and put macrophages into their service to support primary tumor growth.

## Dendritic Cells

Dendritic cells are antigen-presenting cells that elicit innate or adaptive immune responses (Ma et al., 2013). Immature DCs capture tumor-derived antigens and present them on their cell surface to immune cells with proper costimulatory molecules, resulting in an antigen-specific immune response and the formation of T and B cell memories (Ravindran et al., 2019). Nevertheless, DCs exert antitumor or pro-tumor immune responses in accordance with their distinct morphologies and phenotypes.

A growing number of research studies have demonstrated the importance of CSCs in immune evasion by changing DC phenotypes and impeding their recruitment to the TME. CSCs are responsible for influencing the functional differentiation and activation of DCs, turning DCs to become tolerogenic or limiting them to activate T cells (Jachetti et al., 2015; Zhong et al., 2019). CD133^+^ CSCs impair the function of DCs by reducing the quantity of activated DCs in colorectal cancer (Szarynska et al., 2018). The EpCAM^+^ HCC subtype has stemness properties and induces AFP expression, which hinders DC differentiation, maturation and T cell proliferation (Yamashita et al., 2009; Pardee et al., 2014). CSCs also produce immunosuppressive cytokines IL-4, IL-10, IL-13, and TGF-β, and express higher levels of coinhibitory molecules such as PD-L1, B7-H3, and IDO1 (Shipitsin et al., 2007; Todaro et al., 2007). These molecules play crucial roles in accumulating immunosuppressive DCs, which hamper the antitumor response by inducing T cell tolerance and T reg cell recruitment (Boks et al., 2012; Pardee et al., 2014). TGF-β is known for its negative effect on immune response; in terms of DCs, TGF-β inhibits DC activation by suppressing the expressions of its costimulatory molecules CD80 and CD86 and MHC class II (Kobie et al., 2003; Fainaru et al., 2007). Defective RIG-I liver CSCs reduce DC population and induce immunotolerance by upregulating TGF-β signaling (Zhong et al., 2019). Additionally, TGF-β promotes Wnt/β-catenin activation and thus impairs the recruitment of BATF3^+^ DCs, which is correlated with CD8^+^ T cell infiltration (Spranger et al., 2017). Via β-catenin activation, TGF-β impairs T cell mediated immune surveillance and subsides DC recruitment to the tumor site, consequently incurring HCC immune escape and resistance to anti-PD1 treatment (Ruiz de Galarreta et al., 2019). Moreover, TGF-β encourages the development of PD-L1-expressing immunosuppressive DCs, resulting in weakened CD8^+^ T cell activity in a metastatic ovarian cancer model (Cubillos-Ruiz et al., 2010; Krempski et al., 2011).

In the TME, cancer and stromal cells also express C-X-C motif chemokine receptor 4 (CXCR4) and produce its ligand C-X-C motif ligand 12 (CXCL12) to sustain CSC self-renewal and to recruit regulatory DCs. These DCs produce CXCL12 themselves in an autocrine manner and employ a feed-forward mechanism for maintaining CSC stemness (Sultan et al., 2017). Similar to TAM-mediated escape from phagocytic killing, overexpressed CD47 on CSC surface elicits “Don’t eat me” signal by binding to signal regulatory protein alpha (SIPRα), which acts in phagocytosis signaling pathway of DCs (Liu et al., 2017). Although recent findings showed CSCs hijack immune responses by impairing DC functions and recruiting immunosuppressive DC subsets, more investigations are necessary to shed light on the interactions between these two cell types, especially on how DCs alternately regulate CSC stemness properties.

## Myeloid-Derived Suppressor Cells

Myeloid-derived suppressor cells are a heterogeneous subset of myeloid-originated progenitor cells. In humans, these cells are defined by CD11b^+^CD14^–^CD33^+^, while in mice, they are characterized by CD11b^+^Gr1^+^ (Kusmartsev et al., 2004; Nagaraj and Gabrilovich, 2010). MDSCs have been used as a prognostic indicator for patients’ responsiveness to immunotherapy and their survival, as they account for the majority of cells that promote an immunosuppressive environment in the TME (Ai et al., 2018). MSDCs can be classified into two main populations according to their different nuclear morphologies: monocytic-MDSC (mMDSC) and granulocytic-MDSC (gMDSC). They are endowed with different immunosuppressive molecules: mMDSC contains both arginase-1 and iNOS, while g-MDSC contains high levels of arginase-1; therefore, are suggested to exert distinct spatiotemporal regulations on tumor plasticity (Ouzounova et al., 2017). Both mMDSC-derived iNOS and NO, and gMDSC-induced ROS and arginase-1, can lead to TCR peroxynitration and T cell apoptosis (Nagaraj and Gabrilovich, 2010). In addition, MDSCs produce the immunosuppressive cytokines IL-10 and TGF-β as well as PD-L1, which together suppress T cell activity and recruit Tregs (Ostrand-Rosenberg, 2010). They also convey their immunosuppressive functions to macrophages, NK cells and DCs via crosstalk.

Myeloid-derived suppressor cell accumulation in the TME is facilitated by the secretion of cytokines, including IL-1β, IL-6, G-CSF, M-CSF, GM-CSF, macrophage MIF, and TGF-1β, and chemokines CCL1, CCL2, CCL5, CCL22, CXCL2, CXCL5, and CXCL12. The quantity of infiltrating MDSCs is positively associated with CSCs in cancer patients. In a synergistic mammary tumor model, CSCs enhance G-CSF, which is responsible for recruiting MDSCs to the tumor site (Welte et al., 2016). Activation of IL-6/STAT3 signaling has been reported to promote the differentiation of monocytes to MDSCs (Panni et al., 2014). Reciprocally, MDSCs promote the stemness and mesenchymal properties of cancer cells through NOTCH/STAT3 signaling, forming a positive feedback loop with crosstalk between MDSCs and CSCs (Welte et al., 2016; Ouzounova et al., 2017). Via secretion of prometastatic molecules such as MMP9 and chitinase 3–like 1 (CHI3L1), recruited MDSCs enhance stem cell features to promote tumorigenesis and metastasis in triple-negative breast cancer (Kumar et al., 2018). MDSCs also enrich breast cancer cells with stem-like properties by activating IL-6/STAT3 and NO/NOTCH signaling pathways with NO, leading to suppression of T cell activation (Peng et al., 2016). Intriguingly, MDSCs play an additional important role beyond just IL-6-induced transient STAT3 activation. Cell-derived IL-6 further increases IL-6 and IL6Rα in MDSCs, thus allowing MDSCs to prolong STAT3 signaling activation and maintain STAT3 phosphorylation. IL-6-derived MDSC regulation of CSC expansion and immunosuppressive activity is present in both breast and liver cancers (Peng et al., 2016; Xu et al., 2017).

In addition, MDSCs influence cancer stemness via modulation of RNA interference as well as epigenetic regulation. MDSCs trigger miR-101 expression in ovarian cancer, thus inhibit the co-repressor CtBP2 from repressing the transcription of stem cell core genes, leading to an upregulation of stemness markers and tumor growth (Cui et al., 2013). In a co-culture setup, gMDSCs are found to enhance expression of stemness genes and CSC phenotypes of multiple myeloma cell lines through piRNA-823 and subsequent activation of DNA methyltransferases DNMT3B (Ai et al., 2019). MDSCs also increase stem-like properties in ovarian CSCs by upregulating prostaglandin E2 (PGE2) and PD-L1 expressions (Komura et al., 2020). Under hypoxic conditions where liver CSCs are enriched, MDSCs migrate to the tumor site through ENTPD2/CD39 L1 signaling. These MDSCs further promote HCC progression and reduce the efficacy of PD1 therapy (Chiu et al., 2017). Interestingly, depletion of MDSCs leads to sensitization of HCC cells to 5-FU (Xu et al., 2017). Reduction of MDSCs by Listeria bacteria or herpes simplex virus expressing 15-PGDH can attenuate tumor growth and metastasis in breast cancer (Walker et al., 2011; Chandra et al., 2013). All of these findings emphasize the role of MDSCs in reshaping stemness in breast, ovarian and liver cancers and demonstrate the possibility of targeting MDSCs along with CSC eradication in future immunotherapy.

## Regulatory T Cells

Regulatory T cells (Tregs) are a group of CD4^+^ T cells with tumor-promoting effects, usually defined by the Foxp3^+^CD25^+^CD4^+^ T cell subpopulation (Sakaguchi et al., 2010). Tregs abolish host defense mechanisms and exert their functions by inhibiting effector T cells and other immune cells by secreting immunosuppressive cytokines such as IL-10, IL-35, and TGF-β.

A positive correlation has been observed between the presence of CSCs and Tregs in cancers, suggesting possible crosstalk between these cell populations in promoting an immunosuppressive milieu (Yu et al., 2012; Napoletano et al., 2016; Solis-Castillo et al., 2020). In glioblastoma, CSCs induce Treg cell infiltration mediated by the costimulatory molecule PD-L1, soluble Galectin-3, and TGF-β secretion (Wei et al., 2010, 2011), whereas ABCB5^+^ melanoma cells induce Treg cell infiltration via a B7-2-dependent mechanism (Schatton et al., 2010). Chemokines such as CC17, CCL22, and CCL28 are also produced by various cancers to attract Foxp3^+^ Treg cells.

CSCs have been suggested to affect the Th17/Treg balance by altering the production of cytokines such as IL-6 and IL-8 and chemokine CCL5 in the TME (Yu et al., 2012). Treg/Th17 homeostasis has been implicated in its dual effect on the promotion or suppression of cancer (Maniati et al., 2010; Marshall et al., 2016; Knochelmann et al., 2018). A study on Treg and Th17 cells demonstrated STAT3 was a pivotal transcription factor in Th17 differentiation and Treg inhibition, whereas STAT3 is significantly activated in gastric CSCs (Wei et al., 2008; Rezalotfi et al., 2019). Therefore, STAT3 may act as a key factor in modulating CSC stemness and expansion as well as Th17/Treg homeostasis. Yang et al. (2011) demonstrated that IL-17 Tregs stimulate the development of colorectal cancer-related stemness markers, including CD44, CD133, CD166, EpCAM, and ALDH, in bone marrow-derived mononuclear cells and drive cells to become CSCs, indicating the ability of Tregs to induce CSC development. In addition, Tregs release PGE2, which promotes colorectal CSC expansion and metastasis in a mouse model through NF-κB activation (Wang et al., 2015). Indirect interactions between Tregs and CSCs act on the regulation of angiogenesis, TGF-β signaling and macrophage-associated EMT (Mima et al., 2012; Yu et al., 2012; Liu et al., 2021). Under hypoxic conditions, Tregs, which are an important source of VEGF expression, release TGF-β and indirectly regulate CSC expansion by mediating angiogenesis (Facciabene et al., 2011). Additionally, VEGF signaling was found to promote CSC stemness and expansion in melanoma (Beck et al., 2011). Depletion of Tregs lowers VEGF-A and decreases vascularization in tumors. Blockade of VEGFR2 leads to a shrunken CSC population and impaired self-renewal. Similar results have been demonstrated in brain tumors, where the vascular niche directly correlates with CSC generation (Treps et al., 2017). Blockade of angiogenesis signaling significantly inhibits brain CSCs due to reduced blood vasculature in tumors. In line with clinical data, metastatic renal cancer patients who receive antiangiogenic therapy have an overall survival strongly correlated with the reduction in Treg numbers (Brodaczewska et al., 2018). Additionally, the angiogenetic situation is aggravated by TAM preferential secretion of VEGF and IL-8, doubling the effect on promoting CSC proliferation (Werno et al., 2010). Apart from angiogenesis, Tregs also promote CSC expansion by TAM-mediated EMT induction via the expression of CTLA-4, IL-10, and TGF-β (Yu et al., 2012).

Overall, CSCs induce Treg infiltration via costimulatory molecules and STAT3 signaling in the TME, while Tregs alternately regulate CSC proliferation and expansion directly via secretion of IL-17 and PGE2 or indirectly through TGF-β-mediated angiogenesis and EMT.

## Natural Killer Cells

Natural killer cells represent a population of cytotoxic lymphocytes with an innate immune response and are responsible for eradicating tumor cells. High cytotoxic activity of NK cells is correlated with a lowered cancer risk (Imai et al., 2000). Approximately 95% of peripheral blood NK cells are CD56^*dim*^CD16^+^, which exert strong cytotoxic activity.

Beside antibody-dependent cellular cytotoxicity (ADCC) via Fc receptors bound to target cells, NK cells recognize target cells in cell-cell interactions through a variety of activating and inhibitory receptors. Activating receptors, including NKG2C, NKG2D, and NCR, as well as inhibitory receptors, such as Ly49, bind to MHC or HLA class I molecules and cellular stress ligands, leading to the NK cell response (Zhang et al., 2020a). In response to exposure to cancer cells, preferential NK killing of CSCs has been demonstrated in oral squamous carcinoma, human colon carcinoma, melanoma and glioblastoma (Castriconi et al., 2009; Pietra et al., 2009; Tseng et al., 2010; Tallerico et al., 2013; Pan et al., 2015). Specific killing of CSCs with the stem cell markers CD24^+^, CD133^+^, and ALDH^+^ confirms the role of NK cells in effectively targeting and eradicating CSCs. This selective recognition of CSCs has been proposed to be mediated through NKG2D-, DNAM-1- and NKp30-activating receptors (Tallerico et al., 2016). In line with these findings, different types of CSCs express or overexpress the corresponding ligands of those activating receptors with low expression of MHC class I on the surface, leading to effective NK cytotoxicity activity.

However, the preferential tumorigenic capability of CSCs in NOD/SCID mice suggests that there are underlying immunosuppressive mechanisms for CSCs to dodge from NK cell specific killing (Al-Hajj et al., 2003; Tsuchiya and Shiota, 2021). It has been reported that CSCs escape NK-mediated cytotoxicity via various mechanisms by tuning NK receptors. In lung cancer, tumor-derived mesenchymal stem cells (MSCs) alter the NK cell phenotype by downregulating activating receptor expression and inhibiting interferon gamma (IFN-γ) secretion, whereas abortion of PGE2 and restoration of IL-6 activity reverse the tumor-derived MSC-mediated immunosuppression activities (Galland et al., 2017). CD34^+^CD38^–^ leukemic stem cells were shown to be resistant to allogenic NK-mediated killing (She et al., 2012). Breast ALDH^+^ CSCs escape NK cells by reducing the expression of NKG2D ligands MICA and MICB through miR20a modulation (Wang et al., 2014). Downregulation of MICA/B expression supports CSC resistance to NK cell cytotoxicity and increases their metastatic capacity *in vivo*. Recent research also revealed the dual immunoinhibitory role of PCNA in upregulating the stemness of pancreatic and colon CD44^+^CD133^+^ CSCs, as well as participating in immune evasion from NK cytotoxicity by engaging with the inhibitory receptor NKp44 (Malaer and Mathew, 2020). Blockade of the PCNA-NKp44 interaction changes IFN-γ secretion and NK cytotoxicity, suggesting a potential immunotherapeutic target for NK cell-mediated attack. The interaction of NK cell coinhibitory receptors, such as PD-1, with their ligands on tumor cells, also suppresses NK cell-mediated glioma CSC eradication (Huang et al., 2015).

As most NK cell-mediated immune responses occur in tumor cells with low levels of MHC-I, melanoma cancer cells may escape NK cells by upregulating MHC-I on their surface. Interestingly, Huergo-Zapico et al. (2018) suggested that NK cells may release tumor necrosis factor-alpha (TNF-α) and IFN-γ and induce melanoma cells to undergo EMT, pushing them toward invasive phenotypes. EMT induction endows melanoma cells with upregulated stemness markers and enhances their invasive capability. Moreover, EMT favors immune escape by suppressing activating receptors or HLA class-I (Chen et al., 2015). In contrast, some reports have demonstrated that EMT induction promotes NKG2D-L expression on colorectal cells and upregulates NK cell-mediated immunosurveillance in lung cancer (Lopez-Soto et al., 2013; Chockley et al., 2018). This finding suggests that the disparity of the EMT-derived NK cell immune response is dependent on the cancer type.

In summary, NK-mediated killing plays an important role in immune response in diminishing CSCs through the assistance of various activating and inhibitory receptors. Nevertheless, CSCs may escape specific targeting by modulating the expression of these receptors. A novel study also pointed out that NK cells may clash with their classical cytotoxic activity by promoting EMT in CSCs, dependent on the cancer type (Huergo-Zapico et al., 2018).

## Tumor-Infiltrating Lymphocytes

Tumor-infiltrating lymphocytes represent all lymphocytic cell populations, including CD4^+^, CD8^+^, and a small portion of B and NK cells that infiltrate the TME. TILs have been observed in the majority of solid tumors, such as breast, liver and lung cancers (Biller and Dow, 2007). These cells exert diverse effects on the immune response toward the tumor and are correlated with tumor aggressiveness, metastasis, treatment response rate and tumor recurrence. Subsequent to antigen stimulation by APCs, activated helper (CD4^+^) T cells (Th) support the antitumor immune response by further activating cytotoxic (CD8^+^) T cells (CTLs) and recruiting innate immune cells. Th cells stimulate CTLs by IL-2 secretion and cell-cell interactions through costimulatory molecules, including MHC-II, CD27 and CD134 (Giuntoli et al., 2002). Cancer cells, by producing CCL18, recruit Tregs that promote tumor formation and impact other immune cells (Paluskievicz et al., 2019). Bone marrow-derived MSCs have been reported to recruit and maintain Tregs via TGF-β secretion, leading to a negative regulation on T cell proliferation (Di Ianni et al., 2008; Papaccio et al., 2017). Moreover, tumor-derived TGF-β, TNF-α, and IFN-γ induce the differentiation of IL-17^*hi*^ Th17 cells, which supports angiogenesis and enhances protumor transcription factors (Maniati et al., 2010).

The presence of TILs frequently represents a good prognosis for cancer patients (Fridman et al., 2011; Dieci et al., 2014; Idos et al., 2020). Tumor-specific CD8^+^ T cells induced by CSCs *in vitro* demonstrated an effective antitumor response, including inhibiting tumor growth and metastasis with prolonged survival in pancreatic and lung cancer mouse models (Visvader and Lindeman, 2008; Luo et al., 2014). Nevertheless, CSCs are capable of attenuating the action of these cells directly by altering their PD-L1 expression. Elevated stromal TILs and their PD-L1 expression in inflammatory breast cancer and lung adenocarcinoma have been reported to be significantly associated with CSC markers (Mansour et al., 2020; Zhang et al., 2020b). By analyzing PD-L1 expression in a large cohort of HCC patients, Kurebayashi et al. (2018) and others showed that PD-L1 expression in tumor infiltrates is associated with the progenitor subtype of HCC, marked by CK19 and SALL4 expression (Calderaro et al., 2016). High expression levels of PD-L1 are also observed in CD133^+^CD44^+^ colorectal CSCs and CSC-enriched tumor spheres. Hsu et al. (2018) suggested that PD-L1 enrichment in CSCs is mediated by β-catenin/STT3 signaling through glycosylation modulation and PD-L1 stabilization. Based on the clinical correlation between IL-6 and PD-L1 in HCC patient samples, Chan et al. (2019) showed that IL-6 activated JAK1 signaling cascade-induced N-glycosylation and the stabilization of PD-L1. Notch3/mTOR pathway activation is also reported to mediate PD-L1 overexpression on breast CSCs (Mansour et al., 2020). Altered PD-L1 expression, in turn, facilitates colorectal CSC self-renewal with upregulated stemness genes and promotes CSC expansion by activating HMGA1-dependent signaling pathways (Wei F. et al., 2019). PI3K/Akt pathway activation has also been reported to participate in PD-L1-derived promotion of stemness in CSCs (Almozyan et al., 2017).

In addition, interaction with nonlytic CD8^+^ T cells leads to CSC expansion by cell-cell contact in primary breast cancer cell cultures (Stein et al., 2019). The induction of stemness properties in CSCs was confirmed by enhanced tumorigenesis in immunodeficient mice, and the resulting tumors were endowed with a higher cell density and an increased proliferation rate, as well as an elevated chance of lymphoid metastasis. Taken together, these findings showed that the ineffective cytotoxic activity of tumor infiltrates not only fails to eradicate malignancy but also conversely facilitates immune evasion by promoting CSC stemness, proliferation and tumorigenesis of cancer cells. The interaction between various immune cells and CSCs was summarized in Figure 1.

**FIGURE 1:** A diagram illustrating the crosstalk between immune cells and CSCs.

## Development of CSC-Targeted Immunotherapy

Immune checkpoint CTLA-4 and PD-1 inhibitors revolutionized cancer research in the last decade and brought immunology back to the spotlight in therapeutic development. As immunotherapy relies on the immune system to recognize and attack tumor cells, it takes into account not only the tumor cells but also the TME as a therapeutic target to induce a powerful antitumor response. It is clear that CSCs and differentiated tumor cells exhibit distinct gene expression and functions in the tumor bulk, and therefore immunological targeting of the tumor bulk will be biased toward more differentiated tumor cells that express differentiated antigens (Pan et al., 2015). Effective targeting of CSCs may require highly specific identification of the CSC population. Currently, immunological targets of CSCs in therapeutic development have now been focused on three major approaches: CSC-associated antigens, phenotypes and niches.

The innate immune response, including NK and DC cells, exhibits cytotoxic activities toward tumor cells when they are exposed to foreign antigens in the normal immune system. The innate effector and antigen-presenting properties of NK and DC cells empower them to be suitable candidates for immunotherapy. Furthermore, several studies demonstrated that chemotherapy or radiation therapy increased MICA and MICB expression on CSCs, accompanied with CSC expansion (Ames et al., 2015b). This highlights the prospective use of NK cell therapy in combination with traditional therapies in eradicating CSCs. Currently, several clinical trials using NK cells infusion (NCT04162158 and NCT03592706) or in combination therapies (NCT03319459) to treat advanced solid tumors are ongoing. Adoptive NK cell therapy aims to strengthen and reinforce the antitumor functions of NK cells from autologous and allogeneic sources (Wang et al., 2021). After exposure to cytokines such as IL-2 and IL-5, NK cells prolong their activation and exhibit increased cytotoxicity. IL-2- and IL-15-activated NK cells have been shown to be able to eradicate human breast, colon, glioblastoma and melanoma CSCs (Castriconi et al., 2009; Ames et al., 2015a; Yin et al., 2016). A phase I clinical trial using allogeneic NK cells to target CSCs in advanced biliary tract cancer was conducted (NCT03358849). However, the administration of the activating cytokine IL-2 may also lead to the expansion of other immunosuppressive immune cells, including Treg cells (Koreth et al., 2016). In addition, to consistently activate NK cells, the trafficking and maintenance of engineered cytokines such as mbIL-15 and mbIL-21 will also need to be modified during the development of NK cell therapy (Pittari et al., 2015).

Sipuleucel-T is the first FDA-approved DC vaccine against advanced prostate cancer, ensuring DCs as a promising therapeutic strategy in immunotherapy (Cheever and Higano, 2011). DC vaccination has been confirmed to have effective immunologic activities in several preclinical studies. Stimulating DCs with CSC-designated antigens is believed to facilitate CSC eradication with high specificity and effectively resolve CSC-mediated tumor relapse and metastasis (Pang et al., 2019). However, clinical trials reported only a 10 to 15% response to DC vaccination by several cancer types (Anguille et al., 2014). One of the problems leading to low efficacy is the immunosuppressive effect from the upregulation of immune checkpoints (Shi et al., 2018). Recently, CSC-targeted DC vaccines have been reported to enhance the elimination of melanoma CSCs in a mouse tumor model with a combination of PD-L1 and CTLA-4 blockades, with an enhanced CD8^+^ T cell response, increased IFN-γ and inhibited TGF-β expression (Zheng et al., 2018). This finding demonstrates the potential of CSC-based DC vaccines in combinational therapy.

The FDA has approved the use of chimeric antigen receptor (CAR)-T cell therapies targeting CD19 in treating lymphoma since 2017 (FDA, 2017). Increasing numbers of preclinical studies have demonstrated effective immunological control of CAR-T cells in inhibiting cancer growth and prolonging host survival (Chong et al., 2017; Foster et al., 2017; Heczey et al., 2017; Kloss et al., 2018; Zhang et al., 2019). As CAR-T therapy has been in use with a high success rate in treating lymphoma and leukemia, it has also been proposed for targeting CSCs. CSC-related markers such as CD133, EpCAM, and CD90 have been identified as targeted antigens for CAR-T cells (Guo et al., 2018). Zhu et al. (2015) successfully eliminated CD133^+^ CSCs derived from glioblastoma patients; however, T cell aging marker CD57 was induced as a side effect. Recently, a phase I clinical trial (NCT02541370) using autologous CD133-targeted CAR-T cells to treat 23 patients with advanced CD133^+^ tumors resulted in a benefit of 5-month median progression-free survival, with controllable toxicity (Wang et al., 2018b). Zhang et al. (2019) also reported that adoptive transfer of EpCAM-targeted CAR-T cells significantly reduced tumor growth in a xenograft model without safety issues. An EpCAM-targeted CAR-T cell clinical trial (NCT03013712) is in progress for targeting EpCAM^+^ cancers. To minimize the toxicity to normal cells, targeting these CSC markers can be coupled with an inhibitory receptor with specificity for normal tissue antigens.

Yet, more investigations are necessary to overcome the challenges of using CAR-T cells to eliminate CSCs. One of the limitations in developing CAR-T cells targeting CSCs is the diverse treatment response due to the distinct CSCs plasticity and heterogenicity in patients (Alhabbab, 2020). Common immunotherapy hurdles, including acquired resistance as well as upregulation of immune checkpoints are also observed in T cell immunotherapies. Miao et al. (2019) demonstrated that TGF-β-enriched CSCs dampened the cytotoxicity of adoptive T cells by promoting the exhaustion state through CD80-CTLA4 interaction in squamous cell carcinoma. The findings of adaptive immune resistance raised from CSCs against immunotherapy echoes with the previously proposed immunosuppressing feature of CSC, and furthermore emphases CSC as the root of tumor relapse (Tsuchiya and Shiota, 2021).

In addition to direct targeting CSC phenotype and markers, researchers have also targeted the CSC niche, which contributes to CSC self-renewal and immune escape. This includes CSC-associated pathways, cytokines and immune cells (Table 1). As mentioned above, CSCs maintain their self-renewal by generating a positive feedback loop with immunosuppressive cells such as TAMs through JAK/STAT3, Wnt/β-catenin, and NF-κB crosstalk activation, with the expression of inhibitory cytokines such as IL-6, IL-8, and TGF-β. Wnt/ β-catenin-targeted therapies such as anti-FZD receptors monoclonal antibody (Vantictumab), β-catenin inhibitors PRI-724, as well as small-molecule porcupine inhibitor WNT974 are currently in clinical trials. Wnt-targeted treatments are proposed to be implemented as combinational therapies with immune checkpoint inhibitors such as nivolumab and ipilimumab or tyrosine kinase inhibitors, in order to pinpoint the immune evasive ability of CSCs in Wnt-driven cancers (Katoh, 2017). Blockade of IL-6 was previously proven to affect non-small cell lung cancer tumorigenesis and the proliferation of H460 lung CSCs (Yi et al., 2012). The IL-6 receptor monoclonal antibody tocilizumab has been reported to suppress the premetastatic ability of breast CSCs and potentiate the cytotoxicity of cisplatin against triple-negative breast cancer (Alraouji et al., 2020). The drug has been approved by the FDA for treating rheumatoid arthritis and is now under phase II study for curing advanced melanoma in combination with the immune checkpoint inhibitors nivolumab and ipilimumab (NCT03999749). Blockade of the IL-8 receptor CXCR1 using small molecule Reparixin successfully attenuated the CSC population and induced massive apoptosis in a breast cancer cell line. The result of phase I clinical trial showed that Reparixin is safe and well tolerated, in combination of paclitaxel (Schott et al., 2017). Phase II study of this drug showed a ≥20% reduction in CSC markers ALDH^+^ and CD24^–^/CD44^+^ in HER-2-negative breast patients with no serious adverse reactions (Goldstein et al., 2020). Due to the limited number of CSC in primary breast cancer, another clinical trial (NCT02370238) with alternative evaluation endpoint, for example, measurement of metastasis, has been set for assessing the effectiveness of reparixin on CSC eradication (Ruffini, 2019).

**TABLE 1:** Therapeutic strategies targeting the CSC niche and their development progress.

Trial description	Drug name	Moleculartargets	Mechanism of action	Phase of drug development	References
**CSC-associated molecules**					
NK cell therapy		HLA	NK cell killing	I/II	NCT04162158;
				II/III	NCT03592706;
	FAKE-NK100			I	NCT03319459;
	SMT-NK			I	NCT03358849
CAR-T cell therapy	CARTEPC	EpCAM	T cell cytotoxicity	I/II	NCT03013712
		CD133		I/II	NCT02541370
**Pathways**					
iL-6/JAK/STAT	AZD-1480	JAK1/2	Inhibition of JAK1/2	I	NCT01112397
	Celecoxib (FDA approved)	STAT3	Inhibition of STAT3	III	NCT00087256
	Pyrimethamine (FDA approved)	STAT3	Inhibition of STAT3	I/II	NCT01066663
	Tocilizumab	IL-6	IL-6R monoclonal antibody	II	NCT03999749
	Siltuximab	IL-6	IL-6R monoclonal antibody	II	NCT03315026
IL-8	Reparixin	CXCR1	Inhibition of CXCR1	II	NCT01861054;
				II	NCT02370238
NF-kB					
	Acalabrutinib	BTK	Inhibition of BTK	III	NCT04008706
	Ibudilast (MN-166)	TLR4	TLR4 antagonist	II	NCT03782415
	LCL-161	c-IAP	Inhibition of c-IAP	II	NCT01617668;
				I/II	NCT02649673
TGF-β					
	Fresolimumab	TGF-β1/2/3	Neutralizing antibody	II	NCT01472731;
				I/II	NCT02581787
	Galunisertib	TGF-βR1	Inhibition of TGF-βR1	II	NCT02688712;
				II	NCT02538471;
				II	NCT01246986
	Lucanix	TGF-β2	Antisense oligonucleotide	II	NCT01058785;
				III	NCT00676507
	M7824	TGF-β/PD-L1	Ligand trap	III	NCT04066491
Wnt/β-catenin					
	Ipafricept (OMP-54F28)	FZD receptor	FZD8 decoy receptor	I	NCT01608867;
				I	NCT02050178;
				I	NCT02092363;
				I	NCT02069145
	Vantictumab (OMP-18R5)	FZD receptor	Monoclonal antibody against FZD receptors	I	NCT01957007;
				I	NCT01973309;
				I	NCT01345201;
				I	NCT02005315
	PRI-724	CBP/β-catenin	Antagonist	II	NCT01302405
	WNT974	PORCN	Inhibition of PORCN	II	NCT02649530;
				I/II	NCT02278133;
				I	NCT01351103
Notch					
	AL101	γ-Secretase	Inhibition of S3 cleavage	II	NCT03691207
	MK-0752	γ-Secretase	Inhibition of S3 cleavage	I	NCT00106145;
				I	NCT01098344
	Nirogacestat (PF-03084014)	γ-Secretase	Inhibition of S3 cleavage	II	NCT02109445;
				II	NCT02299635
	Demicizumab (OMP-21 M18)	DLL4	Blockade of DLL4	II	NCT02259582
	Enoticumab (REGN421)	DLL4	Monoclonal antibody against DLL4	I	NCT00871559
VEGF					
	Axitinib	VEGFR	Inhibition of VEGFR	I	NCT02853331
	Bevacizumab (FDA approved)	VEGFR	Inhibition of VEGF binding to receptor	II	NCT02226289;
				III	NCT02420821;
				III	NCT03434379
**Immune cells**					
TAMs	Zoledronate acid	Mevalonate pathway	Elimination	I/II	NCT00588913;
				III	NCT02622607
	BMS-813160	CCR2/5	Inhibition of macrophage recruitment	II	NCT04123379;
				I/II	NCT03767582;
				I/II	NCT03496662;
				II	NCT02996110
	BL-8040	CXCR4	Antagonist	II	NCT02826486;
				II	NCT02907099
	Pexidartinib	CSF-1R	Inhibition of CSF-1R	I	NCT02777710
	AMG820	CSF-1R	Monoclonal antibody against CSF-1R	I/II	NCT02713529
	ALX148	CD47/SIRPα	Blockade of CD47	I	NCT03013218
	IBI322	CD47/SIRPα	CD47/PD-L1 bispecific antibody	I	NCT04328831
	Hu5F9-G4	CD47/SIRPα	Monoclonal antibody against CD47	I	NCT02216409
MDSCs	INCB001158	Arginase	Inhibition of arginase	I/II	NCT02903914
	Decitabine	Arginase	Differentiation	I	NCT00030615
	Entinostat	Arginase	Elimination	I	NCT02453620
NK cells	Lirilumab	KIR	Blockade of inhibitory signal of NK cells	I/II	NCT03532451;
					NCT01714739
	Monalizumab (IPH2201)	NKG2A	Inhibition of immune checkpoint	I/II	NCT03822351;
					NCT03833440
Tregs	Ontak (Denileukin diftitox)	CD25	Induction of apoptosis	II	NCT00726037

The roles of angiogenesis in supporting immunosuppressive TME and self-renewal of CSCs have been extensively studied, thus the combination use with VEGF inhibitor provides a novel direction for immunotherapy. A phase III clinical trial (NCT03434379) of bevacizumab with PD-L1 inhibitor atezolizumab showed a superior outcome in overall and progression-free survival than sorafenib in advanced HCC cases (Finn et al., 2020). Due to this encouraging result, FDA approved the combined use of bevacizumab and atezolizumab as the first-line treatment for unresectable HCC patients (Yang et al., 2020). A recent report on targeting aberrant mRNA modification in leukemia has highlighted another potential therapeutic approach to suppress fat mass and obesity-associated protein (FTO), an RNA N6-methyladenosine (m6A) demethylase (Su et al., 2020). M6A RNA modification has been implicated in self-renewal and tumorigenesis in various cancers, thus is proposed to be a novel therapeutic target against CSCs (Ma and Ji, 2020). Using small molecule inhibitors CS1 and CS2, inhibition of FTO attenuates self-renewal ability of leukemic stem cells via reducing MYC and CEBPA expressions. Targeting FTO also suppresses the immune checkpoint gene LILRB4, and thus sensitizes the cancer cells to T cell cytotoxicity (Su et al., 2020). Thus, the combination of FTO inhibitors and hypomethylating agents (HMA) is recommended for future clinical trials, in order to overcome the adaptive immune resistance induced by HMA treatment in leukemia patients with high FTO.

Direct targeting of immunosuppressive cells such as TAMs with zoledronic acid successfully inhibited the growth of cervical cancer cell-derived CSCs by reducing their stemness properties and inducing apoptosis (Wang et al., 2019). The drug is now undergoing phase III clinical trials to examine its preventive effect on bone metastasis in patients with advanced lung cancer (NCT02622607). CD47-targeting antibodies also overcome a key immune escape mechanism, the CD47/SIRPα-mediated “Don’t eat me” signal. ALX148, which is a CD47 blocking protein, was well tolerated in combination with anticancer antibodies and conventional chemotherapy in patients with advanced cancers (NCT03013218). Hu5F9-G4, an anti-CD47 antibody, also shows excellent tolerability and promising effects in leukemia stem cells in combination with Azacitidine (NCT03248479). These findings suggest that targeting CD47 with conventional cancer treatment may be a powerful strategy to address CSC-derived immune evasion. Ontak, a fusion protein comprized of human IL-2 and diphtheria toxin, targets CD25^+^ Treg cells by inducing apoptotic cell death (Cheung et al., 2019). A pilot study was carried out to evaluate its inhibitory effect on Tregs in metastatic pancreatic cancer patients (NCT00726037). This drug is designed to integrate DC vaccine administration for treating unresectable pancreatic cancer. Several clinical trials aiming at other immunotherapeutic targets, such as MDSCs and NK cells, are also ongoing (Table 1).

While direct CSC-targeted treatments such as NK, CAR-T therapies and DC vaccines are still being studied, targeting the CSC niche might be a feasible immunological therapeutic approach to eradicate cancer, considering several encouraging preclinical results. Similarly, much effort will be required to resolve the side effects such as the resistance or diverse treatment responses that most immunotherapies may arouse. Additionally, basic research on the crosstalk between CSCs and their niche is also necessary for identifying a biomarker that can monitor the treatment response, as well as novel therapeutic targets for the development of effective treatments.

## Author Contributions

ML: conception and design, writing, review, and/or revision of the manuscript. TL: study supervision. Both authors contributed to the article and approved the submitted version.

## Conflict of Interest

The authors declare that the research was conducted in the absence of any commercial or financial relationships that could be construed as a potential conflict of interest.

## Abbreviations

ADCC: antibody-dependent cellular cytotoxicity
CSC: cancer stem cell
CCL: C-C motif chemokine ligand
CAR: chimeric antigen receptor
CHI3L1: chitinase 3–like 1
CXCR: C-X -C motif chemokine receptor
CXCL: C-X -C motif ligand
CTL: cytotoxic T cell
CTLA-4: cytotoxic T-lymphocyte -associated protein-4
DC: dendritic cell
EMT: epithelial–mesenchymal transition
FTO: fat mass and obesity-associated protein
HCC: hepatocellular carcinoma
HMA: hypomethylating agents
IFN- γ: interferon gamma
gMDSC: granulocytic MDSC
IL: interleukin
MSC: mesenchymal stem cell
mMDSC: monocytic MDSC
MDSC: myeloid-derived suppressor cell
m6A: N6-methyladenosine
NK: natural killer
NF- κ B: nuclear factor- κ B
NFAT: nuclear factor of activated T-cells
PD-1: programmed cell death protein
PD-L1: programmed death-ligand 1
PGE2: prostaglandin E2
Siglec-10: sialic-acid-binding Ig-like lectin 10
SIPR α: signal regulatory protein alpha
STAT3: signal transducer and activator of transcription 3
TIM-3: T cell immunoglobulin and mucin domain-containing protein-3
Th cell: T helper cell
TGF- β: transforming growth factor beta
Treg: T regulatory
TAM: tumor associated macrophage
TIL: tumor-infiltrating lymphocyte
TME: tumor microenvironment
TNF- α: tumor necrosis factor-alpha
VEGF: vascular endothelial growth factor.
